# The Outcome and Safety in Laparoscopic Common Bile Duct Exploration with Primary Suture versus T-Tube Drainage: A Meta-Analysis

**DOI:** 10.1155/2023/7300519

**Published:** 2023-02-07

**Authors:** Xianhua Ma, Shengbin Cai

**Affiliations:** ^1^Oncology Ward, Dushu Lake Hospital Affiliated to Soochow University, Medical Center of Soochow University, Suzhou Dushu Lake Hospital, Suzhou 215123, Jiangsu, China; ^2^General Surgery Ward, Dushu Lake Hospital Affiliated to Soochow University, Medical Center of Soochow University, Suzhou Dushu Lake Hospital, Suzhou 215123, Jiangsu, China

## Abstract

**Background:**

Sometimes, after choledochotomy, the common bile duct is closed with T-tube drainage for several weeks to prevent postoperative complications such as biliary fistula and stricture. But there has been controversy over the advantages of primary suture versus T-tube drainage. The purpose of our meta-analysis in laparoscopic common bile duct exploration is to appraise the efficacy and safety of T-tube drainage and primary suture.

**Methods:**

The literatures were searched by Web of Science, PubMed, Cochrane Library, OVID, and EMBASE between the year January 1, 2001 and February 28, 2021. Meta-analysis was performed by Stata 12.

**Results:**

Fourteen studies with 1,549 patients (827 vs. 722) were included in our study. The primary suture group had significant lesser operative time (*P* ≤ 0.001), postoperative hospital stay (*P* ≤ 0.001), hospital expenses (*P* ≤ 0.001), intraoperative bleeding (*P*=0.001), and postoperative complications (*P*=0.006) than the T-tube drainage group. In postoperative bleeding (*P*=0.289), bile leakage (*P*=0.326), and bile duct stricture (*P*=0.750), there was no statistical difference. In the primary suture group, using single-arm synthesis, the bile leakage rate and the bile duct stricture rate were 0.07 vs. 0.04 and 0.00 vs. 0.00 in interrupted suture and continuous suture groups. The bile duct stricture rate was same in both groups, and the bile leakage rate was lower in the interrupted suture group. But the difference was not significant.

**Conclusion:**

The primary suture group had several advantages, including lesser operative time, postoperative complications, intraoperative bleeding, postoperative hospital stay, and hospital expenses. In bile leakage and bile duct stricture, the difference between the two groups was not significant. In the primary suture group, interrupted suture and continuous suture groups had similar bile leakage rate and bile duct stricture rate.

## 1. Introduction

Common bile duct (CBD) stone is a common complication of cholelithiasis that appears during the natural history of this entity [1]. Of individuals with symptomatic gallstones, CBD stone is estimated to be present in 10%–20% [2], which is associated with cholangitis, jaundice, acute pancreatitis, and other serious complications [3], and can have serious consequences caused by these. For choledocholithiasis, based on refinements in laparoscopic technique and operative skills and the development of instruments, laparoscopic common bile duct exploration (LCBDE) has become more and more popular and feasible. Ordinarily, after choledochotomy and removal of CBD stones, the CBD is closed with T-tube drainage (TD) for several weeks to prevent postoperative complications such as biliary fistula and stricture. Therefore, patients must carry it for several weeks before removal, which significantly reduce the quality of patients' life. However, T-tube usage is not without morbidity. These problems led some surgeons to try to perform laparoscopic primary duct closure after choledochotomy. Therefore, after LCBDE, there has been controversy over the advantages of primary suture (PS) versus TD. The purpose of our research is to compare the safety and efficacy of TD and PS for the CBD stones treatment.

## 2. Materials and Methods

### 2.1. Search Strategy

We conducted this study according to the Preferred Reporting Items for Systematic Reviews and Meta-Analyses (PRISMA) statement. Related articles were searched by two authors in Web of Science, PubMed, OVID, Cochrane Library, and EMBASE using the following keywords: “laparoscopic common bile duct exploration,” “primary suture,” and “T-tube drainage.” We also reviewed the references of included articles to identify additional studies. All studies published between the year January 1, 2001 and February 28, 2021. Languages were limited to English and Chinese. Most studies are carried on in China.

Inclusion criteria were as follows:

1. All patients were diagnosed with choledocholithiasis
2. The PS group received LCBDE with primary closure
3. The TD group underwent LCBDE followed by TD

Exclusion criteria were as follows:

1. Incomplete data
2. Duplicate studies
3. Based on animals or nonhuman samples
4. Case reports or reviews

### 2.2. Data Extraction

Two reviewers separately performed the search, then reviewed the titles, abstracts, and full texts of all studies, and extracted the following data from each eligible study. Author, publication year, study type, inclusion and exclusion criteria, subjects' number, and the evaluation index included operative time, postoperative hospital stay, intraoperative bleeding, hospital expenses, postoperative complications, postoperative bleeding, bile leakage, and bile duct stricture were collected from each study.

### 2.3. Quality Assessment

The modified Jadad method was used to measure the quality of randomized controlled trial (RCT). Studies awarded four or more points were defined as high-quality studies. The quality of nonrandomized studies was assessed by the Newcastle–Ottawa Scale (NOS) [4], and <4 stars were considered as low quality, 4–6 stars as medium quality, and >7 stars as high quality.

### 2.4. Statistical Analysis

Stata 12 was used for meta-analysis. Heterogeneity among the studies was analyzed by chi-square test and *I*^2^ test. *P* < 0.05 and *I*^2^ > 50% were considered as statistically significant heterogeneity and a random-effects model was selected. Otherwise, a fixed-effects model was selected. Dichotomous data were calculated by odds ratio (OR) and 95% confidence interval (95% CI), whereas continuous data were calculated by weighted mean difference (WMD) and 95% CI. Probability value of *P* < 0.05 was considered statistically significant. Single-arm meta-analyses were performed to evaluate bile leakage and bile duct stricture rates for continuous suture (CS) and interrupted suture (IS) in PS group. Begg's test was used to assess publication bias.

## 3. Results

### 3.1. Base Characteristics

One-hundred ten studies were identified; 38 studies were excluded after duplicate removal. After examining the titles and abstracts, we excluded 48 articles. After full-text article review, 10 studies were excluded. Finally, 14 articles [5–18] were enrolled for analysis, including 1,549 patients: 827 and 722 patients are in PS and TD groups (Figure 1). The patients' data are listed in Table 1.

### 3.2. Meta-Analysis Results

#### 3.2.1. Operative Time

The operative time was provided in nine articles. The random-effects model was used because significant heterogeneity was found (*I*^2^ = 73%, *P* ≤ 0.001). The PS group had a lesser operative time than the TD group, and the difference between the two groups was significant (WMD = −26.98, 95% CI (−33.14, −20.82), *P* ≤ 0.001) (Figure 2).

#### 3.2.2. Intraoperative Bleeding

The intraoperative bleeding was reported in five articles. High heterogeneity was observed (*I*^2^ = 68.8%, *P*=0.012). Therefore, we used the random-effects model. Our study points out that the intraoperative bleeding in the PS group was lesser, and the difference was statistically significant (WMD = −7.92, 95% CI (−12.45, −3.39) *P*=0.001) (Figure 3).

#### 3.2.3. Postoperative Hospital Stay

Ten articles reported the postoperative hospital stay. The random-effects model was used because of the high heterogeneity (*I*^2^ = 75.1%, *P* ≤ 0.001), and our meta-analysis showed that compared with the TD group, the PS group had a lesser postoperative hospital stay (WMD = −2.40, 95% CI (−2.92, −1.88), *P* ≤ 0.001) (Figure 4).

#### 3.2.4. Hospital Expenses

The hospital expenses were reported in five Chinese studies. Significantly high heterogeneity was observed (*I*^2^ = 96.3%, *P* ≤ 0.001), thus the random-effects model was chosen. The study showed that the PS group had lower hospital expenses than the TD group (WMD = −2675.18, 95% CI (−3785.18, −1565.17), *P* ≤ 0.001) (Figure 5).

#### 3.2.5. Postoperative Complications

Nine studies reported postoperative complications. There was no heterogeneity observed between these studies (*I*^2^ = 0.0%, *P*=0.917). Hence, we selected the fixed-effects model. The meta-analysis showed that the postoperative complications in the PS group were lower than the TD group, and the difference between the two groups was statistically significant (OR = 0.58, 95% CI (0.39, 0.85), *P*=0.006) (Figure 6).

#### 3.2.6. Postoperative Bleeding

The postoperative bleeding was provided in six studies. There was no heterogeneity between these studies (*I*^2^ = 0.0%, *P*=0.989), so the fixed-effects model was selected. In the postoperative bleeding, there was no significant difference between the PS group and the TD group (OR = 0.48, 95% CI (0.12, 1.86), *P*=0.289) (Figure 7).

#### 3.2.7. Bile Leakage

The bile leakage was reported in 14 articles. In the fixed-effects model (*I*^2^ = 0.0%, *P*=0.795), there was no statistically significant difference in the bile leakage (OR = 1.26, 95% CI (0.79, 2.00), *P*=0.326) (Figure 8). Among them, there are four articles of CS and five articles of IS in the PS group. The remaining five articles either did not specify the suture method or mixed the two suture methods in the PS group. In single-arm synthesis, the bile leakage was 0.07 (95% CI 0.02–0.13) and 0.04 (95% CI 0.02–0.06) in CS and IS groups. The bile leakage rate was lower in the IS group; however, the difference was not statistically significant (Figure 8).

#### 3.2.8. Bile Duct Stricture

Nine articles reported the bile duct stricture and showed that there was no significant difference in the bile duct stricture between the two groups (OR = 1.55, 95% CI (0.19, 12.46), *P*=0.679). There was no heterogeneity observed (*I*^2^ = 0.0%, *P*=0.499), therefore the fixed-effects model was selected (Figure 9). Among them, there are four articles of CS and four articles of IS in the PS group. The remaining one article mixed the two suture methods. In single-arm synthesis, the bile duct stricture was 0.00 (95% CI 0.00–0.03) and 0.00 (95% CI 0.00–0.00) in CS and IS groups. The bile duct stricture rate was same in two groups, and the difference was not significant (Figure 9).

#### 3.2.9. Publication Bias

Begg's test demonstrated that there was no potential publication bias.

## 4. Discussion

In gallstone patients, CBD stone is a common disease with an incidence rate of 10%–20% [19], which is associated with acute suppurative cholangitis, obstructive jaundice, acute pancreatitis, and other serious complications. Traditionally, after LCBDE, the CBD is closed with TD. Temporary TD is usually required because of papilla edema caused by stone extraction, increasing the pressure inside the biliary tree [20]. The advocates argue that it relieves spasm or edema of sphincter after the trauma caused by the exploration [10] and prevents bile stasis, biliary fistula, and stricture, and decompresses the biliary tree and removal of residual stones. Nevertheless, insertion of TD has several complications, such as increasing the patients' psychological pressure, difficulty in nursing after discharge, accidental displacement of the TD, and biliary leakage. After discharge, patients have to carry the TD for several weeks, requiring continuous management and restricting patient activity, which have extremely reduced the quality of life of patients. Therefore, some surgeons try to operate LCBDE with primary closure.

Over the years, a lot of surgeons have contrasted LCBDE with and without TD. Many researchers are worried about postoperative biliary leakage and bile duct stricture after the primary closure. Therefore, they choose to place TD. Since first used by Kehr [21], the TD has been used to prevent biliary leakage and bile duct stenosis after choledochotomy for over 100 years. But, with the increase in laparoscopic experience and the improvement in the laparoscopic devices and instruments, LCBDE with PS became more and more widely practiced. Particularly, choledochoscope usage ensures direct visualization of the CBD and enables its complete clearance and exploration of the distal CBD [7]. But there still has been huge controversy over the advantages of TD versus PS. So, we conducted this meta-analysis to contrast the safety and efficacy of TD and PS for CBD stones.

Based on our meta-analysis, the PS group had a significantly lesser operative time (WMD = −26.98, 95% CI (−33.14, −20.82), *P* ≤ 0.001) and intraoperative bleeding (WMD = −7.92, 95% CI (−12.45, −3.39) *P*=0.001). The longer operating time for the TD group may be caused by the complexity of the surgery, such as TD insertion. Wu et al. [22] found that longer anesthesia and operation time may be related to an increased thromboembolic risk and cardiac and respiratory complications. Postoperative complications in the PS group were significantly lower (OR = 0.58, 95% CI (0.39, 0.85), *P*=0.006), and postoperative hospital stay (WMD = −2.40, 95% CI (−2.92, −1.88), *P* ≤ 0.001) is also lower in the PS group. Length of hospital stay may be affected by open T-tube risk factors, such as dehydration, electrolyte disorder, displacement of drainage tube, and localized pain. Lower postoperative complications and postoperative hospital stay led lower hospital expenses (WMD = −2675.18, 95% CI (−3785.18, −1565.17), *P* ≤ 0.001). But surgeons are concerned about postoperative biliary leakage and bile duct stricture after the primary closure. Based on our study, there was no significant difference in the bile leakage (OR = 1.26, 95% CI (0.79, 2.00), *P*=0.326) and the bile duct stricture (OR = 1.55, 95% CI (0.19, 12.46), *P*=0.750) between the two groups. This means that PS does not increases bile leakage and bile duct stricture rates.

Ordinarily, there are now two kinds of suturing methods, namely, IS and CS. There still has been no conclusion about which suture method is better. Therefore, in the PS group, we used single-arm meta-analysis to compare the bile leakage and bile duct stricture rates after using IS and CS. In single-arm synthesis, the bile leakage rate was 0.07 (95% CI 0.02–0.13) and 0.04 (95% CI 0.02–0.06) in CS group and IS group. The bile leakage rate was lower in the IS group. The bile duct stricture rate was 0.00 (95% CI 0.00–0.03) and 0.00 (95% CI 0.00–0.00) in both groups. The bile duct stricture rate was same in the two groups. But the difference was not significant in both the bile leakage rate and the bile duct stricture rate.

The research by Wang et al. [8] shows that compared with T-tube group, PS reduces immunologic suppression. Surgical trauma causes alterations in the systemic immune response. Placement of TD, which is a foreign body, can increase white blood cell (WBC) and interleukin-6 (IL-6) levels and also suppress tumor necrosis factor-*α* (TNF-*α*). The operative time in TD group is longer than PS group, which may strengthen the immune response. Furthermore, placement of TD also increases the patients' psychological pressure, causes pain, and reduces the quality of life of patients. These factors may damage the immune function to some degree, thereby increasing the possibility of fever, infection, and other complications.

We acknowledge that there are some limitations in our study. First, more than half of included studies are non-RCT studies. Second, sample size is too small in some studies, especially in single-arm meta-analysis in bile leakage rate and the bile duct stricture rate. Third, although postoperative complications, postoperative bleeding, bile leakage, and bile duct stricture have no heterogeneity, other outcomes such as operative time, intraoperative bleeding, postoperative hospital stay, and hospital expenses have high heterogeneity. Some factors, such as surgical experience, surgical instruments, and different discharge standards, may have explained the high heterogeneity. But these might have affected the results. Therefore, larger, well-designed, multicenter, high-quality, randomized controlled clinical trials should be performed to confirm the results.

## 5. Conclusion

In this meta-analysis, we have observed that, although postoperative bleeding, bile leakage, and bile duct stricture did not differ significantly, patients in the PS group had better outcomes, such as operative time, intraoperative bleeding, postoperative hospital stay, hospital expenses, and postoperative complications, than those in the TD group. In the PS group, the bile duct stricture rate was same in the IS group and the CS group, and the bile leakage rate was lower in the IS group. But the difference was not statistically significant between the two groups.

## Figures and Tables

**Figure 1:** Flow diagram of study screening and inclusion.

**Figure 2:** Forest plot and funnel plot of the operative time between the primary suture group and the T-tube drainage group.

**Figure 3:** Forest plot and funnel plot of the intraoperative bleeding between the primary suture group and the T-tube drainage group.

**Figure 4:** Forest plot and funnel plot of the postoperative hospital stay between the primary suture group and the T-tube drainage group.

**Figure 5:** Forest plot and funnel plot of the hospital expenses between the primary suture group and the T-tube drainage group.

**Figure 6:** Forest plot and funnel plot of the postoperative complications between the primary suture group and the T-tube drainage group.

**Figure 7:** Forest plot and funnel plot of the postoperative bleeding between the primary suture group and the T-tube drainage group.

**Figure 8:** Forest plot of meta-analysis and single-arm meta-analysis and funnel plot of the bile leakage between the primary suture group and the T-tube drainage group.

**Figure 9:** Forest plot of meta-analysis and single-arm meta-analysis and funnel plot of the bile duct stricture between the primary suture group and the T-tube drainage group.

**Table 1:** Characteristics of the included studies.

First author	Year	Study design	Total cases	No. of patients (primary suture: T-tube)	Included outcomes	Quality
Zhou	2019	Retrospective	79	38:41	a, b, c, e, f, g, h	8
Cai	2012	Retrospective	239	137:102	a, b, c, e, f, g, h	8
Wang	2014	Prospective	240	132:108	a, b, c, f, g, h	9
Parra-Membrives	2017	Retrospective	88	36:52	e, g, h	7
El-Geidie	2010	RCT	122	61:61	e, f, g	5
Zhang	2017	Retrospective	78	38:40	a, c, g	7
Tang	2013	Retrospective	105	85:20	a, c, d, f, g, h	8
Wang	2013	Retrospective	71	39:32	e, g	8
Zheng	2017	Retrospective	67	34:33	a, b, c, g	7
Ha	2004	Retrospective	38	12:26	e, g, h	7
Leida	2008	RCT	80	40:40	c, d, e, g, h	6
Zhang	2008	RCT	93	47:46	a, c, d, e, g	6
Dong	2014	RCT	194	101:93	a, b, c, d, e, g, h	6
Zhang	2004	RCT	55	27:28	a, c, d, e, g, h	4

Included outcomes: a, operative time; b, intraoperative bleeding; c, postoperative hospital stay; d, hospital expenses; e, postoperative complications; f, postoperative bleeding; g, bile leakage; h, bile duct stricture.

## Data Availability

The datasets generated and/or analyzed during the current study are available in Web of Science, PubMed, OVID, Cochrane Library, and EMBASE. The datasets used and/or analyzed during the current study are available from the corresponding author on reasonable request.

## Abbreviations

CBD: Common bile duct
LC: Laparoscopic cholecystectomy
LCBDE: Laparoscopic common bile duct exploration
ERCP: Endoscopic retrograde cholangiopancreatography
TD: T-tube drainage
PS: Primary suture
PRISMA: Preferred Reporting Items for Systematic Reviews and Meta-Analyses
RCT: Randomized controlled trial
NOS: Newcastle–Ottawa Scale
OR: Odds ratio
WMD: Weighted mean difference
CI: Confidence interval
CS: Continuous suture
IS: Interrupted suture.
